The article "Study on the Expression Profile of Autophagy-Related Genes in Colon Adenocarcinoma" was published in 2022. Journal: Comput Math Methods Med.

# Study on the Expression Profile of Autophagy-Related Genes in Colon Adenocarcinoma

**DOI:** 10.1155/2022/7525048

**Published:** 2022-05-04

**Authors:** Mingyu Hou, Jiakang Ma, Jun Ma

**Affiliations:** ^1^Department of Oncology, The Second Affiliated Hospital, Zhengzhou University, Zhengzhou, 450014 Henan, China; ^2^Institute of Digestive Disease, Zhengzhou University, Zhengzhou, 450014 Henan, China

## Abstract

Colon adenocarcinoma (COAD) is a common digestive tract tumor. Autophagy-related genes (ARGs) may play an obbligato role in the biological processes of COAD. This study was aimed at exploring the role of ARGs in COAD. Clinical data and RNA sequencing data of tumor and healthy samples were obtained from The Cancer Genome Atlas (TCGA), and discrepantly expressed ARGs were screened. Statistical differences of ARGs were performed with Gene Ontology (GO) functional annotation and the Kyoto Encyclopedia of Genes and Genomes pathway enrichment analysis. Eight ARGs were selected by univariate Cox and multivariate Cox regression. Kaplan–Meier (K-M) and multivariate receiver operating characteristic (multi-ROC) were used to check the fitness of the model. Among 398 COAD samples and 39 normal samples obtained from the TCGA database, 37 differentially expressed ARGs were screened. In the training group, eight prognostics-related ARGs (MTMR14, VAMP3, HSPA8, TSC1, DAPK1, CX3CL1, ATG13, and MAP1LC3C) were identified by Cox regression. A gene signature risk prediction model was constructed base on 8 autophagy-related genes. The survival time of the low-risk group was longer than the high-risk group, and the AUC of the model was 0.794. Univariate and multivariate Cox regression analysis showed that age and riskscore were the independent predictor. In conclusion, the prognosis model we built based one ARGs of COAD patients can estimate the prognosis of patients in clinical treatment.

## 1. Introduction

Colon cancer is a widely known tumor, and its incidence rate is increasing. Epidemiological studies have shown that approximately 10% of all cancer deaths is caused by colon cancer and related complications [1]. Colon adenocarcinoma is the most common, accounting for 98% of colon carcinoma cases [2]. Colon cancer has a high recurrence rate after treatment, 42% of patients will relapse within 5 years, and the median time from recurrence to death is 12 months [3]. In addition, the molecular mechanism of colon cancer is still unclear. Therefore, we decided to explore the molecular mechanism of COAD.

Autophagy is an important metabolic process that occurs only in eukaryotic cells. It enables lysosomes to decompose abnormal, dysfunctional proteins and organelles and can provide nutrients and energy for cells [4]. In previous studies, autophagy has been found to be involved in multiple physiological processes, especially closely related to cell death, and involved in many signaling pathways. There are sufficient evidences that autophagy can promote or inhibit tumor growth through Bcl-2, EGFR, and other signaling pathways [5]. Research by Catalano et al. shows that ARGs upregulated two master regulators of epithelial-mesenchymal transition (EMT), SNAIL, and SLUG, to promote EMT [6]. Zeng and Ju's study suggested that autophagy guided by the Hedgehog signaling pathway leads to tumor cell death [7]. Sandilands's team found that SRC's autophagy targeted at focal adhesion kinase (FAK) signaling promotes cancer cell survival [8]. These studies suggest that autophagy may promote tumor occurrence and progression through a variety of signaling pathways.

The article "Study on the Expression Profile of Autophagy-Related Genes in Colon Adenocarcinoma" was published in 2022. Journal: Comput Math Methods Med.

Scientists have done a lot of research on the role of autophagy in tumors. Some studies have shown that autophagy can block tumor production. Peng et al.'s team found that BECN1 (encoding BECN1/Beclin 1), which induces autophagy, is cleaved and inactivated by caspase-3 in the absence of an abhydrolase domain containing 5 (ABHD5); ABHD5 increases the genomic instability and promotes the occurrence of cancer [9]. De et al. found that autophagy can inhibit angiogenesis by inducing endothelial cell death, thus inhibiting tumor growth indirectly [10]. However, other studies have found that autophagy promotes tumor genesis and growth. A study by Wen et al. showed that autophagy enhanced fatty acid utilization by tumor cells and caused adipocytes' growth-promoting effect blocked. In this study, fatty acid activates autophagy in colon cancer cells and promotes tumor cell growth [11]. A study has shown that RACK1 promotes the reproduction of colon carcinoma cells by inducing autophagy and enhances the viability of them [12]. The recurrence of ovarian tumors after dormancy induced by ARHI tumor suppressor also depends on autophagy [13]. Zhao et al.'s team found that autophagy can enhance the invasiveness of prostate cancer [14]. Some studies confirmed that the autophagy phenomenon is related to tumor resistance and metastasis [15]. Sharifi et al. revealed that autophagy plays a significant role in tumor cell migration. Autophagy defective tumor cells cannot decompose focal adhesion and metastasis [16]. Some studies have confirmed that autophagy can inhibit metastasis of tumor cells. Gugnoni et al.'s team has shown that autophagy can inhibit EMT and cancer metastasis, which can be blocked by cadherin-6 [17].Therefore, it is very important to explore molecular biomarkers suitable for the clinical treatment and prognosis of colon cancer. Liu et al. [18] constructed on 13 ARG-based prognostic model using information obtained from the TCGA and HADb databases and finally identified 3 high-risk genes, namely, MAP1LC3C, RAB7A, and WIPI2, as prognostic biomarker genes for CRC.

The article "Study on the Expression Profile of Autophagy-Related Genes in Colon Adenocarcinoma" was published in 2022. Journal: Comput Math Methods Med.

In general, considering the contradictory and complex role of autophagy genes in COAD, the novelty and motivation of this study is to explore the law of COAD autophagy by analyzing the ARG expression and corresponding clinical information of the Cancer Genome Atlas (TCGA) database. First, ARGs with differential expression levels in tumor and normal tissues were screened out, and the possible pathways of ARGs were explored by Gene Ontology (GO) functional enrichment and the Kyoto Encyclopedia of Genes and Genomes (KEGG) pathway annotation. Then, Cox regression was used to determine which ARGs are associated with the prognosis of COAD patients and used to construct the model. To test the model accuracy, the Kaplan–Meier (K-M) method and the receiver operating characteristic (ROC) curve was plotted.

## 2. Materials and Methods

### 2.1. Data Acquiring and Preprocessing

A total of 232 ARGs found from the Human Autophagy Portal (http://www.autophagy.lu/index HTML) contain all the ARGs in the human genome. RNA sequencing and clinical records of 398 tumor samples and 39 healthy samples were extracted from the TCGA database. The data used in the GO enrichment comes from the Cistrome project (http://www.cistrome.org/). The data used in the KEGG enrichment comes from the KEGG project (http://www.kegg.jp/).

### 2.2. Choosing Discrepantly Expressed ARGs in COAD

The ARG expression of 398 tumor samples and 39 normal samples was averaged, and the limma package of R language was used to analyze the expression difference of each gene in tumor and normal samples. The threshold is ∣log2 fold change (FC) > 1, and adjusted *P* value <0.05. Next, we integrated the discrepant data of expressed ARGs in tumor and healthy colon tissues with their corresponding clinical information for further analysis.

### 2.3. Enrichment Analysis of ARGs

To investigate the potential tumor-associated molecular mechanism of ARGs, we used the R language to annotate the GO function and the enrichment analysis of the KEGG pathway. The R package includes Goplot, DOSE, ggplot2, enrichplot, clusterProfiler, and BiocManager, with a *P* value of 0.05. The formula of the *Z*-score is $Z-\text{score}=\sqrt{U-D/T}$, where *U* represents upregulated genes enriched in GO, *D* represents downregulated genes enriched in GO, and *T* means the number of genes enriched in the pathway.

### 2.4. Construction of the Prognostic Model

The 38 ARGs with differential expression in COAD tissues and normal tissues were analyzed by univariate Cox regression, and 24 ARGs were found to be significantly related to prognosis (*P* < 0.05). Then, we used a multivariate Cox analysis to adjust the gene parameters in each model to avoid overfitting. The remaining eight ARGs were elements to construct the prognosis model.

The article "Study on the Expression Profile of Autophagy-Related Genes in Colon Adenocarcinoma" was published in 2022. Journal: Comput Math Methods Med.

The risk calculation method of the ARG model is Riskscore = ∑_*i*=1_^*n*^*v*_*i*_*c*_*i*_,

where *v*_*i*_ represents the expression of the gene *i*, *c*_*i*_ is the regression coefficient of the gene *i* calculated by multivariate Cox regression analysis, and *n* represents the total number of independent indicators.

### 2.5. Verify the Accuracy of the Model

Based on the median risk score of samples, we divided the patients into low-risk and high-risk groups. K-M survival curve was used to evaluate the statistical divergence between the two groups. We also used the ROC curves to test the fitting of the model.

### 2.6. Statistical Analysis

Strawberry Perl (http://strawberryperl.com/) was used to organize data. R4.0.2 (https://www.r-project.org/) was used for most statistical analysis and graphic rendering. K-M curve was drawn to describe the diversity of survival rate in high-risk group and low-risk groups. The fitting performance of the model was evaluated by the area under the curve (AUC) of the multi-ROC curve. The statistical graphs and statistical information of genes and clinical traits in the model are provided by UALCAN (http://ualcan.path.uab.edu/). The statistical charts of model risk score and clinical parameters are drawn by SPSS26.0.

## 3. Results and Discussion

### 3.1. Expression of ARGs in COAD and Normal Tissues

Whether autophagy can lead to cell death is related to the level of autophagy-targeting compounds, Allison S. Limpert believes that excessive levels of autophagy have been shown to promote autophagy-dependent cell death. We analyzed the gene expression in 398 COAD samples and 39 normal samples by the Wilcoxon Signed-Rank Test. 37 differentially expressed ARGs were identified from 232 ARG according to the criteria of ∣ log2FC  | >1 and adjusted *P* value < 0.05 (Figure 1). Among them, 21 were low expression (HSPB8, NKX2-3, NRG2, TP53INP2, CCR2, TMEM74, NRG3, MAP1LC3C, BCL2, PINK1, FKBP1B, TNFSF10, NRG1, ITPR1, PRKN, FAS, SESN2, GABARAP, FAM215A, CAPN2, and CDKN1A) in tumor tissues, and 16 were high expression (MBTPS2, CAPN10, BCL2L1, ERO1A, BID, ATIC, HSP90AB1, CD46, EIF4EBP1, BIRC5, VEGFA, SPHK1, MYC, TP73, CDKN2A, and ATG9B) in tumor tissues. The expressions of 37 ARGs in tumor and normal tissues are shown in Figure 1(c).

### 3.2. GO and KEGG Analyses of ARGs

To explore the molecular mechanism of ARGs in the oncogenesis of COAD, we conducted GO functional annotation and KEGG pathway enrichment analysis on ARGS. The results of GO enrichment showed that ARGs mainly participated in autophagy, dealing with changes in oxygen content and intrinsic apoptotic signaling pathways in biological processes (BP). In cellular components (CC), it is mainly focused on autophagosome and vacuolar membrane. The molecular function (MF) is mainly responsible for ubiquitin kinase regulator activity and protein ligase binding (Figures 2(a) and 2(b)). In KEGG enrichment analysis, ARG mainly participates in the signaling pathway of P53 and erbB, apoptosis, drug resistance of platinum, and EGFR tyrosine kinase inhibitor and participates in human cytomegalovirus infection (Figure 2(c)).

The article "Study on the Expression Profile of Autophagy-Related Genes in Colon Adenocarcinoma" was published in 2022. Journal: Comput Math Methods Med.

### 3.3. Survival-Associated ARGs and the Prognostic Model

The biomarkers of gene sequencing can directly deduce the survival time of colon carcinoma patients, independent of tumor-node-metastasis stage [19]. Through univariate Cox regression analysis, 24 ARGs associated to the survival rate of COAD patients were identified (Figure 3), of which 8 (MTMR14, VAMP3, HSPA8, PRKAB1, BIRC5, BID, ATG3, and MAP1LC3C) were negatively correlated with risk score and 17 (GABARAP, HSPB8, TSC1, PEA15, DAPK1, PELP1, CDKN2A, CX3CL1, GRID1, ATG13, SPHK1, ZFYVE1, CFLAR, MAP1LC3C, MAP2K7, ULK1, and CTSD) were positively correlated with risk score (*P* < 0.05).

### 3.4. Model Construction

According to the eight candidate ARGs, the model for the risk score of COAD patients was built with gene expression value (GEV): risk score = (GEV of MTMR14∗−1.57825) + (GEV of VAMP3∗−0.50804) + (GEV of HSPA8∗−0.41769) + (GEV of TSC1∗0.76707) + (GEV of DAPK1∗0.31191) + (GEV of CX3CL1∗0.26684) + (GEV of ATG13∗0.73431) + (GEV of MAP1LC3C∗2.272704981).

The results illustrated that patients in the low-risk group survive longer than the high-risk group. We also calculated and ranked patients' risk score by the model (Figures 4(a) and 4(b)). The scatterplot also shows that patients in the low-risk group survive longer than the high-risk group (Figure 4(c)). The results of expression level of genes in different risk group revealed that high-risk patients have a lower content of MTMR14, VAMP3, and HSPA8 in colon tissue than low-risk patients, and content of TSC1, DAPK1, CX3CL1, ATG13, and MAP1LC3C is on the opposite (Figure 4(d)).

### 3.5. Model Performance Verification

To verify the fitting degree of the model, we also examined the relationship between model elements and clinical risk, and the forest map shows the association between risk factors and prognosis (Figures 5(a) and 5(b)). We also drew the K-M curve to inspect the survival of two risk groups, and the results showed that high-risk patients were significantly associated with poor outcomes (Figure 5(c)). The AUC of the model ROC curve is 0.794 (Figure 5(d)).

The article "Study on the Expression Profile of Autophagy-Related Genes in Colon Adenocarcinoma" was published in 2022. Journal: Comput Math Methods Med.

### 3.6. The Correlation between Model Elements and Clinical Parameters of COAD

The relationship between riskscores of model and clinical parameters of COAD is shown in Figures 6(a) and 6(c), and the results revealed that riskscores have statistically significant correlation to clinical parameters of COAD. In addition, in model elements, statistical differences were showed in the expression of HSPA8 and TSC1 in COAD based on nodal metastasis status (Figures 6(d) and 6(f)), as well as the expression of HSPA8 and VAMP3 in COAD based on individual cancer stages (Figures 6(e) and 6(g)).

## 4. Discussion

COAD is the major subtype of colon cancer in histology. COAD cannot be effectively prevented, attributed to the large number of patients and deaths caused by COAD [1, 20]. There is a lot of evidence indicating that autophagy is involved in multiple BP of COAD. Studies have shown that cryptotanshinone guides autophagic cells death through ROS-p38 MAPK-NF-*κ*B signaling pathway [21]. Wen et al. found that orexin-A induced autophagy of colon cancer cells through extracellular signal-regulated kinase (ERK) signaling pathway, thus hindering the reproduction of colon carcinoma cells [22]. Yan et al. found that the inhibition of 6-phosphofructo-2-kinase/fructose-2, 6-bisphosphatase isoform 3 (PFKFB3) attenuated oxaliplatin-induced autophagy and decreased the viability of colon cancer cells [23]. Son et al. observed that the inhibition of autophagy of HCT116 in colon cancer cells by 3-MA could increase the rate of apoptosis [24].

In present research, we examined the ARG expression profiles of COAD samples in the TCGA database and found that 37 ARGs had statistical difference between tumor and normal tissues. We performed GO and KEGG enrichment analyses on the discrepantly expressed ARGs. In addition to the autophagy pathway, these ARGs were also related to the BP of oxygen level responses. Azad et al. believed that the reactive oxygen species (ROS) could induce autophagy, low levels of ROS induced autophagy can inhibit tumor apoptosis, but excessive ROS will cause tumor cell death, and high levels of ROS will cause cancer [25]. In this study, we found that the autophagy-related proteins of COAD are distributed in autophagy bodies and also in vacuoles, both of which are important places for autophagy [26–28]. As for the function of MF, ARGs are mainly enriched in protein kinase regulator activity and ubiquitin-protein ligase binding. This binding is the main pathway of protein degradation that plays an indispensable role in autophagy. Protein kinase regulator activity can activate proteins to participate in various BP. In KEGG enrichment, ARGs are concentrated in signaling pathways of p53 and erbB, apoptosis, platinum drug resistance, and EGFR tyrosine kinase inhibitor and concentrated in human cytomegalovirus infection. P53 is an important tumor suppressor gene. It has been reported that TP53-HMGB1 complexes in the cytoplasm can regulate the balance between autophagy and apoptosis. Apoptosis occurs when there are more TP53 in the cytoplasm, and autophagy occurs when there is more HMGB1 [29]. The enrichment of ARGs in platinum drug resistance suggests that platinum drug resistance in colon cancer may be related to autophagy. The prognostic model constructed in this study involves eight proteins, namely, MTMR14, vesicle-associated membrane protein 3 (VAMP3), HSPA8, TSC1, DAPK1, CX3CL1, ATG13, and MAP1LC3C. As far as we know, this is also the first time that MTMR14 and VAMP3 were found to play a role in COAD. It is reported that the loss of MTMR14 can cause autophagy disorder and lead to muscle disease [30, 31]. The validated VAMP3 is generally regarded as a kind of biomarker of cell aging associated with multiple kinds of tumors, such as pancreatic cancer and breast cancer [32], and can reduce cell invasiveness [33].

The article "Study on the Expression Profile of Autophagy-Related Genes in Colon Adenocarcinoma" was published in 2022. Journal: Comput Math Methods Med.

TSC1 is an important part of the survival promoting PI3K/Akt/mTOR signaling pathway. By cooperating with a variety of regulatory molecules, TSC1 plays an important role in development, cell growth and proliferation, survival, autophagy, and ciliary development [34]. TSC1/TSC2 tumor suppressor complex can be used as an inhibitor of mTOR pathway. The destruction of TSC1/TSC2 tumor suppressor function may contribute to the occurrence of tumor [35]. It is reported that low TSC1 expression level is associated with poor clinical outcomes of breast cancer [36] and gastric cancer [37]. Meanwhile, the nanoscale effects of some proteins we have found associated with autophagy and colon cancer have been studied. Nanoparticulate titanium dioxide can downregulate the expression of TSC1 in mouse follicles [38]. At the same time, nanoparticulate titanium dioxide can induce podocyte autophagy through antioxidant mechanism [39]. Nanoliquid chromatography tandem mass spectrometry suggested that HSPA8 might be related to pregnancy [40]. Microcapillary reverse-phase high-performance liquid chromatography-nanoelectrospray tandem mass spectrometry showed that VAMP3 was a factor involved in the secretion of platelet granules [41]. This evidence suggests that our model will be more valuable in scientific research when deeply combined with nanotechnology. More studies have proved that nanotitanium dioxide has tremendous potential in the treatment of colon adenocarcinoma. TSC1 is a kind of oncogene in colon cancer. Using nanotitanium dioxide to reduce the expression of TSC1 in colon cancer cells may become a new method for the treatment of colon cancer. Studies have shown that titanium dioxide nanoparticles can inhibit tumor cells by stimulating oxidative stress [42]. However, nano-TiO2 has a wide range of biological effects, which is deleterious to multiple organs in mammals [43]. Proquin et al. found that titanium dioxide nanoparticles may cause canceration of normal colon cells [44]. Therefore, it will be a research direction to make nano-TiO2 specifically combine with tumor cells.

The article "Study on the Expression Profile of Autophagy-Related Genes in Colon Adenocarcinoma" was published in 2022. Journal: Comput Math Methods Med.

There are some deficiencies in our research. First, the molecular mechanism speculated in this study has not been verified by experiments. Second, the model of this study has not been applied in clinical settings, and its effect has not been confirmed. In addition, the specific molecular mechanisms of eight kinds of ARGs need to be further studied.

## 5. Conclusion

The purpose of this research is to penetrate the role of ARGs in COAD and construct a prognostic model of COAD patients with ARGs, which can be used as a method for the prognosis of COAD patients. We also identified the pathways involved in ARGs related to the occurrence of COAD, which can be used to study the role of autophagy in COAD.

## Figures and Tables

**Figure 1:** Differentially expressed ARGs in COAD. (a) Heat map presenting the difference in the expression of ARGs between COAD and normal specimens. Red represents a high expression of ARGs in tissues, and green means low expression. (b) Volcano maps of 232 ARGs. Red represents genes that are highly expressed in tumor tissues, while green represents genes with low expression. (c) The expression of different ARGs in COAD.

**Figure 2:** GO and KEGG pathway enrichment analysis of ARGs. (a) The number of genes enriched in each GO. (b) *Z* − score > 0 indicates more upregulated genes enriched in this pathway, and vice versa. (c) KEGG pathway enrichment analysis of ARGs.

**Figure 3:** The forest map shows the hazard ratio of ARGs. Red indicates that the expression of ARGs is positively correlated to patients' survival, and the green represents that ARGs are negatively correlated to patients' survival.

**Figure 4:** The riskscore, survival time, and survival status of the prediction model. (a) Expression of ARGs in the model in two groups. (b) The prognostic model distribution of COAD patients. (c) COAD patients' survival in the TCGA dataset. (d) The expression level of genes in difference risk group. ^∗∗∗^*P* < 0.001.

The article "Study on the Expression Profile of Autophagy-Related Genes in Colon Adenocarcinoma" was published in 2022. Journal: Comput Math Methods Med.

**Figure 5:** Verification of the model. (a) Analysis of univariate independent prognostic showed the association between risk factors and prognosis. (b) Results of multivariate independent prognostic showed the association between risk factors and prognosis. (c) Survival curve calculated by the model. (d) Multi-ROC of each risk factor.

**Figure 6:** Model elements which have statistically significant correlation to clinical parameters of COAD. (a) The relationship between riskscore and nodal metastasis status. (b) The relationship between riskscore and nodal metastasis status. (c) The relationship between riskscore and individual cancer stages. (d) The relationship between HSPA8B and nodal metastasis status. (e) The relationship between HSPA8B and individual cancer stages. (f) The relationship between TSC1 and nodal metastasis status. (g) The relationship between VAMP3 and individual cancer stages (*P* < 0.05).

## Data Availability

We would like to thank the TCGA team, Cistrome project team, KEGG project team, and UALCAN team for allowing us to use their data. The objects of this study are publicly available datasets. The datasets are excerpted from the TCGA database, Cistrome project (http://www.cistrome.org/), and KEGG project (http://www.kegg.jp/). The statistical graphs and information on genes and clinical traits in the model are provided by UALCAN (http://ualcan.path.uab.edu/).
